# Biologically Derived Gold Nanoparticles and Their Applications

**DOI:** 10.1155/2022/8184217

**Published:** 2022-08-01

**Authors:** Arpita Roy, Chetan Pandit, Amel Gacem, Mohammed S. Alqahtani, Muhammad Bilal, Saiful Islam, Md. Jamal Hossain, Mohammed Jameel

**Affiliations:** ^1^Department of Biotechnology, School of Engineering & Technology, Sharda University, Greater Noida, India; ^2^Department of Life Sciences, School of Basic Sciences and Research, Sharda University, Greater Noida, India; ^3^Department of Physics, Faculty of Sciences, University 20 Août 1955, BP26 21000, Skikda, Algeria; ^4^Radiological Sciences Department, College of Applied Medical Sciences, King Khalid University, Abha 61421, Saudi Arabia; ^5^BioImaging Unit, Space Research Centre, University of Leicester, Michael Atiyah Building, Leicester LE1 7RH, UK; ^6^School of Life Science and Food Engineering, Huaiyin Institute of Technology, Huai'an 223003, China; ^7^Civil Engineering Department, College of Engineering, King Khalid University, Abha 61421, Saudi Arabia; ^8^Department of Pharmacy, State University of Bangladesh, 77 Satmasjid Road, Dhaka, Bangladesh; ^9^Department of Civil Engineering, College of Engineering, King Khalid University, Abha, Saudi Arabia

## Abstract

Nanotechnology is a rapidly evolving discipline as it has a wide variety of applications in several fields. They have been synthesized in a variety of ways. Traditional processes such as chemical and physical synthesis have limits, whether in the form of chemical contamination during synthesis operations or in subsequent applications and usage of more energy. Over the last decade, research has focused on establishing easy, nontoxic, clean, cost-effective, and environmentally friendly techniques for nanoparticle production. To achieve this goal, biological synthesis was created to close this gap. Biosynthesis of nanoparticles is a one-step process, and it is ecofriendly in nature. The metabolic activities of biological agents convert dissolved metal ions into nanometals. For biosynthesis of metal nanoparticles, various biological agents like plants, fungus, and bacteria are utilized. In this review paper, the aim is to provide a summary of contemporary research on the biosynthesis of gold nanoparticles and their applications in various domains have been discussed.

## 1. Introduction

Nanotechnology is an evolving area due to its wider range of applications in a variety of disciplines [1, 2]. Optics, electronics, catalysis, biomedicine, magnetics, mechanics, and energy research are some of the fields where nanotechnology is applied [3]. Nanobiotechnology is a collaborative area that entails technology research and development in a variety of domains such as nanotechnology, biotechnology, chemistry, material science, and physics [4]. It is about the biofabrication of nano-objects or bifunctional macromolecules that may be utilized to produce or modify nano-objects [5]. Nanoparticles are metallic units that come in a variety of forms, including spherical, triangular, and rod shaped [6]. Nanoparticles have distinct features (chemical, physical, optical, and so on) as compared to bulk material [7]. Currently, research on nanoparticles production is one of the hot topics.

One of most well-defined noble metals is gold. It is utilized in automobiles as a heat insulator and as a reflective coating on some high-end CDs [8]. Gold nanoparticles (GNPs) are being researched for usage in ultrasensitive chemicals, optoelectronic devices, or biological sensors, or as catalysts [9]. Among all types of nanomaterials, metallic nanoparticles are the most promising because of their excellent antibacterial characteristics due to their huge surface area to volume ratio. Researchers are interested in the antibacterial effect of metallic nanoparticles because of the rising microbial resistance to antibiotics or the creation of resistant strains. Silver, platinum, gold, titanium, iron, palladium, aluminum, and copper [10] are some of the metallic nanoparticles that have received a lot of attention recently owing to their critical value. Gold has been used in medicine in various forms throughout the history of civilization. Rheumatic illnesses, such as discoid lupus erythematosus and restorative dentistry, and different skin inflammation conditions, such as urticaria, pemphigus, and psoriasis, have been treated with gold and gold compounds [11].

Biological agents such as plant tissues, bacteria, fungi, actinomycetes, and other molecules have been used for synthesis of gold nanoparticles. The extracellular synthesis of gold nanoparticles has attracted a lot of interest because it avoids many stages of the synthesis process. In general, there are two techniques for nanoparticle synthesis, that is, a ‘top-bottom' and a ‘bottom-top' strategy. Nanoparticles could be synthesized by chemical (chemical reduction) or biological (uses of plant, microbes, etc.) processes through self-assembly of atom new nuclei that develop into nanoscale particles in the bottom-top approach [12]; however, in the top-bottom method, appropriate bulk materials are reduced into small particles using different lithographic processes. Physical and chemical processes for nanoparticle synthesis are not environmentally friendly due to the usage of toxic substances that pose a variety of biological dangers and are costly [13]. This review provides a summary of contemporary research on biosynthesis of gold nanoparticles and their applications in various domains.

## 2. General Chemistries of Gold

There are six possible oxidation states for gold, ranging between −1 and +5, due to its comparatively high electronegativity. Auric (Au (I)) or auric (Au (III)) are two of the main oxidation states for gold complexes [14]. To dissolve gold in aqueous solution, the oxidation and complexation processes work together. Au (I) or Au (III) could form a stable complex in the presence of complex ligands, or, in solution, these could be reduced to metals of gold. Stabilities of gold's complex is governed not just by complex ligand's property, but also by the donor atom of ligands which is directly attached to gold atoms [15]. The first rule, according to research, is that stability of gold's complex reduces as the electronegativity of the donor atom rises. In solution, the stability of the gold halide complex, for example, follows the I- > Br- > Cl- > F patterns [16]. The second rule is that Au (III) is preferred to Au (I) in harsh ligands, whereas Au (I) is preferred to Au (III) in gentle ligands (III). Preferred coordination numbers of Au (I) are 2, which results in a linear complex, whereas Au (III) has a preferred coordination number of 4, which results in a square planar complex. Two precursor uses in the production of GNPs are the gold (III) chloride complexes or the gold thiosulfate (I). In most GNP biosynthesis techniques, the gold (III) chloride complexes are extensively employed as precursors.

## 3. Green Synthesis of Gold Nanoparticles

One of the basic and technical concerns is the production of nanoscale gold within the regulated phase or shapes. Michael Faraday described production of gold colloids, now known as GNPs, nearly 150 years ago using phosphorous to decrease AuCl4 ions. A variety of biological, physical, or chemical methods have been explored in the past years in order to create GNPs for usage in electrical, biotechnological, industrial, pharmaceutical, agricultural, or medical sectors [17]. These methods are used to manufacture gold nanostructures with well-defined compositions, such as colloids, clusters, wires, powders, tubes, rods, and thin films [18]. Physical and chemical approaches to make GNPs have been used in the past, as shown in Figure 1. These approaches have yielded GNPs within size ranging from 1 to 100 nm or varieties of morphology. These synthesis processes have certain limitations despite their considerable research, such as the use of harsh chemicals, rigorous synthesis conditions, energy or capital demands [19], or lower productivities [20]. Currently, mix-shaped nanoparticles (NPs), produced by synthetic methods, need high-cost, low-yield purification processes such as differential centrifugation [6]. Furthermore, these processes create more sludge and pose environmental risks due to harmful solvents or additives. As a result, there is a growing need to create clean, nontoxic, ecologically friendly, and long-term synthesis methods. A key issue is the development of high-yield, low-cost NPs production technologies. Because of their wide range of applications, researchers in nanoparticles synthesis had turned to a biological system.

Biosynthesis has been shown to be a viable method for producing tiny particles on a wide scale [21] (Figure 2). It is worth noting that biologically produced NPs have higher stability [23] and better morphological control. Biological systems that create NPs include bacteria, fungus, actinomycetes, and plants [24, 25]. Microbes create NPs intracellularly and/or extracellularly due to their inherent potential [26]. However, due to the further processing procedures, such as ultrasonication or treatments with appropriate detergents, extracting NP generated via intracellular biosynthesis is often challenging [27]. As a result, bacteria that produce NP extracellularly must be thoroughly screened [28]. Microorganisms as potential biofactories for GNP production is a promising new field of study. Additionally, it can easily be scaled up for larger-scale production and is economical, time-saving, and ecologically friendly [29]. Next sections go through the various microbial synthesis techniques for GNPs in further depth.

### 3.1. Bacteria

Prokaryotes have gained a lot of interest in the field of GNP synthesis among microorganisms. For the first time, bacterial generation of GNP in *Bacillus subtilis* 168 was described, indicating the presence of 10–35 nm octahedral NPs in the cell wall [30]. *Rhodopseudomonas capsulata* generated spherical GNPGNP within diameters of 10–20 nm at a lower concentration [31] or nanowires within networks at high concentrations [32]. In a study, GNP synthesis has been reported in six cyanobacteria which include *Plectonema* sp.*, Calothrix* sp.*, Anabaena* sp., and *Leptolyngbya* sp. GNP [33]. Govindaraju et al. [34] reported synthesis of GNPs from single celled protein, that is, *Spirulina platensis* GNP.  Table 1 summarizes the synthesis of bacterial GNP. Ahmad et al. [44] demonstrate microbial generation of monodispersed GNPs from an extremophilic *Thermomonas* sp. A study reported that after 48 hours of incubation with aqueous chloroauric acid (HAuCl_4_) solution at pH ranges of 4.0–7.0, bacterium *Rhodopseudomonas capsulata* produces spherical GNPs in 15–25 nm ranges [31]. Furthermore, pH of the solution is an important factor that influences types of biogenic AuNPs or location of gold deposition in the cell. Due to metal ion reduction by enzyme present in cell walls or on the cytoplasmic membrane but not in the cytosols, alkalotolerant *Rhodococcus* sp. formed more intracellular monodispersed GNPs on the cytoplasmic membrane than on the cell walls. *Pseudomonas aeruginosa* cell supernatant was used for the reduction of gold ions and extracellular production of GNPs [36]. Heterotrophic sulphate-reducing bacteria were employed in the bacterial cell membrane to decrease gold (I) thiosulfate complexes Au (S_2_O_3_)_2_ to elementals golds of 10 nm sizes, resulting in H2S as a metabolic end product [48]. *E. coli* DH5 biologically reduces chloroauric acid to Au0, leading to the synthesis of nanoparticles on the cell surface, which were mostly spherical but also included some triangles or quasihexagons. This cell-bounded nanoparticles might be useful in hemoglobin or protein electrochemistry [49]. *Rhodobacter capsulatus*, a photosynthetic bacterium with a larger biosorption capacities for HAuCl_4_, have also been found to bioreduce trivalent aurum. Carotenoid or NADPH-dependent enzyme incorporated in plasma membranes or released extracellularly had been identified to have a role in biosorption or bioreduction of Au^3+^ to Au^0^ both inside and outside cells [50].

### 3.2. Fungi

Fungi are among the most effective microbial agents for the production of metal nanoparticles. *Fusarium oxysporum, Trichothecium* sp.*, Colletotrichum* sp.*, Trichoderma asperellum, Phanerochaete chrysosporium, T. viride, Fusarium semitectum, Coriolus versicolor, Aspergillus fumigates,* or *Phoma glomerata* are examples of fungi. Fungi are believed to be more advantageous for GNP synthesis than other bacteria because fungal-mycelial meshes, unlike bacteria, could withstand flow pressure, agitations, or other bioreactor conditions. They are easy to culture and manage. They produce more reductive protein extracellular secretions and are more easily processed downstream [51]. Fungus *Trichothecium* sp. was reported to produce GNPs both extracellularly and intracellularly [52]. Under stationary conditions, gold ion interacting within *Trichothecium* sp. fungal biomass results in rapid extracellular formations of GNPs with spherical rod-like and triangular shapes, whereas in case of shaking condition it resulted in intracellular formation of the GNPs. A study reported that whenever gold ions are exposed to extremophilic actinomycete *Thermomonospora* sp., it reduces metal ions extracellularly [53].  Table 2 provides an overview of fungal derived GNP production.

### 3.3. Plant

One of the most significant methods for biosynthesis of nanoparticles was the use of plant extracts (Figure 3). In a study, *Azadirachta indica* leaf extract showed bioreduction of Au^3+^ or Ag^+^ ion [69]. Aloe vera leaf extract was used to make gold nanotriangle and spherical silver nanoparticles [70]. Some of the ecological benefits of processing plants or their extracts in producing GNPs include uses of nontoxic biocomponents to cap or reduce GNP, limiting waste generation, eliminating the need for further purification methods or ease of availability. Flavonoids, phytosterols, quinones, and other plant biocomponents contribute to the formation of GNPs because they include functional groups that aid in the reduction and stability of GNPs. To create specified shapes and sizes of GNPs, technique requires the combination of gold salt with plant extracts for a certain period of time under various reaction variables such as pH, incubation duration, and temperature.

Song et al. [71] reported GNPs synthesis from leaf extract of two plants, that is, *Magnolia kobus* and *Diospyros kaki*. GNPs were synthesied by using a plant extract mixed with an aqueous HAuCl4 solution. At a reaction temperature of 95°C, more than 90% of the GNPs were recovered in just a few minutes. *Emblica officinalis* fruit extract was also used as a reducing agent in extracellular synthesis of extremely stables Ag nanoparticles [72]. In a study, *Cinnamomum camphora* leaf extract was used to make gold nanoparticles [73]. Further information on the plants that have been used for synthesis of GNPs has been provided in Table 3.

### 3.4. Algae

Algae is one of the potential biological agents which can be utilized for the synthesis of different types of nanoparticles. There is a current interest in the study of algal mediated synthesis of metal nanoparticles, with a focus on the evaluation of the effect of reaction conditions, such as pH, temperature, and stirring rate, upon the final nanoparticles with respect to size, morphology, stability, and so forth [102]. A study employed algal system to explore procedure of gold's reduction by *Chlorella vulgaris* biomass from gold (III) chloride solution [103]. XAS data show that Au (III) was significantly reduced to Au (I), also Au (I) is coordinated along sulfur atom from free-sulfhydryl residue or lighter-atoms elements, most likely nitrogen. Another study reported that elemental gold was largely precipitated on cell wall of *Sargassum natans* biomass [104]. According to a study, hydroxyl groups of saccharide or carboxylates anions of amino acid residues from peptidoglycans layers on cell walls seemed to be the gold binding site [105]. A marine alga *Sargassum wightii* was also used for production of GNPs [106]. After 12 hours of reaction, stable GNPs in the size range of 8–12 nm was produced through reducing aq. AuCl4- ions within extracts of marine alga, with 95% of golds recovered. Some other algae which are used for the synthesis of gold nanoparticles include *Acanthophora spicifera*, *Kappaphycus alvarezii, Chlorella pyrenoidosa*, *Sargassum myriocystum*, *Stoechospermum marginatum*, *Sargassum wightii*, and *Laminaria japonica* [107]. Arockiya Aarthi Rajathi et al. [108] reported synthesis of gold nanoparticles using *Stoechospermum marginatum* and the synthesized nanoparticles were 18.7–93.7 nm in size. Another study reported synthesis of gold nanoparticles using *Tetraselmis kochinensis* with 5–35 nm in size [109]. Abdel-Raouf et al. [110] reported synthesis of gold nanoparticles using Galaxaura elongata with the size range of 3.85–77.13 nm. *Sargassum cymosum* synthesized gold nanoparticles were reported by Costa et al. [111] with the size range of 7–20 nm.

### 3.5. Biomolecules

Biomolecules are molecules that are produced by living organisms to help the body's biological processes. Some of the biomolecules include amino acids, nucleic acids, carbohydrates, and lipids. Carbonyl and hydroxyl groups of biomolecules convert Au^3+^ ion to Au^0^ atom. After that, Au^0^ is capped, yielding stable GNPs. The biosafety of the reactants employed in the manufacture of GNP's may be addressed using this technique.  Table 4 depicts the various biomolecule-mediated GNP production methods. List of different biomolecules which were utilized for gold nanoparticles synthesis has been reported in Table 4.

## 4. Advantages of Biologically Synthesized Gold Nanoparticles

Biogenic gold nanoparticles are free from hazardous by-products which are generally found in case of chemical synthesis, that resulted in minimising usage in different applications [128]. To be used in biomedical applications, gold nanoparticles must be biocompatible. Biological production of gold nanoparticles had various advantages, including its simplicity, one-step nature, environmental friendliness, cost effectiveness, and biocompatibility [129]. Furthermore, no external stabilising agents are required since biogenic components of plants and microorganisms serve as stabilising or capping agents. Biosynthesis of gold nanoparticles requires less time than chemical one. Another advantage of biological synthesis is that it could decrease numbers of chemical synthesis steps required, such as adding functional groups to surfaces of gold nanoparticles to make them physiologically active [129].

## 5. Applications of GNPs

The productions of inorganic or metal-based nanomaterials had encouraged establishment of newer industry which brings together experts from several sectors to hunt for new type of nanoparticles having distinct property. Developing or designing creative or cost-effective processes for scaling up the nanomaterial manufacturing has not only given an intriguing topic of research but will also address future human needs such as health, safety, and environmental concerns. Nanomaterials are rapidly being used in industry, also these would soon replace hazardous or toxic chemical usage. The utilization of nanoparticles or nanocomposites is relatively safer option, opening up new areas for antibacterial research. Different ancient cultures (India, China, or Egypt) employed gold to heal diseases like smallpox, syphilis, skin ulcers, or measles [130].

### 5.1. Medical Application

Gold nanoparticles are versatile materials with several uses in a wide range of industries. Gold particles were coated with DNA and inserted into plant embryos or plant cells by researchers. This ensures that some genetic material enters and transforms the cells. This technique improves plant plastids. Because GNPs may be detected using a number of methods, including optical absorptions fluorescent or electrical conductivities, they had been mainly used in biosensor labelling and bioimaging applications [131]. GNPs were focused and amplified in regions of interests, giving contrasts for observations or visualisations. Light energy causes free electrons in GNPs to form collective oscillations *k*/*a*, a surface plasmon, which has the property of considerably absorbing and scattering visible light. The excited electron plasma thermally relaxes by the transfer of energies to gold lattices, causing GNPs to heat up as a result of light absorption. The interaction of GNPs with light can assist in optical microscopy, fluorescent microscopy, photothermal imaging, or photoacoustic imaging. In addition, transmission-electrons microscopy [132] may be used to investigate interactions of GNPs with electrons wave or X-ray. Gold nanoparticles have long been used to carry therapeutic compounds into cells [133]. Before being administered to cells by gene guns or particle ingestion, the chemicals are adsorbed on the surface of GNPs.

#### 5.1.1. Anticancer Activity

GNPs are used to treat cancer because of their biocompatibility. GNPs might be utilized to treat epithelial ovarian cancer. They have the capacity to suppress the evolution of ovarian cancer and metastasis [134]. Growth factors VEGF (vascular-endothelial growth factors) are involved in the development of ovarian cancer and tumour growth. GNPs have also been demonstrated to inhibit activity of VEGF, which promotes cell proliferation, in multiple myeloma (MM), a plasma cell cancer. As a result of VEGF inhibition, cell-cycle inhibitor proteins such as p21 or p27, that limit proliferations, are upregulated [135]. Chronic lymphocytic leukaemia (CLL) is a kind of leukaemia characterised by an excess of lymphocytes that originate in bone marrow but could spread to different organs. GNPs have been found to inhibit the action of factor produced by CLL cells or to promote apoptosis [136] because they have the potential to impair the function of heparin-based growth factors.

#### 5.1.2. Tumour Detection

Newly developed functionalized GNPs (dendrimers) have been developed to target and destroy tumours and combat cancer [137]. GNPs are intended not only to recognise, target, and destroy tumours, but also to transport an additional chemical that can delay or kill cancerous cells. Dendrimers function as arm for GNPs, allowing other molecules to be attached to the arms. Laser and infrared light heat gold's particle, prompting dendrimer in releasing chemicals that kill tumours. The Mie equations suggest that the surface plasmon resonance scattering of GNPs will increase as the nanoparticle size grows. By conjugating GNP to anti-EGFR antibodies, using stronger scattering images of GNP coupled to antibodies which just adhere to cancerous cells and not to noncancerous cells, researchers were able to distinguish between cancerous and noncancerous cell [138]. A basic optical microscope is used to view the scattering. They obtain 500% greatest bindings ratios to sick cells compared to nonmalignant cells, allowing cancerous cells to be spotted using a dark field microscope to examine scattered light. Because of their higher X-ray's absorption coefficient, simplicity of synthetics modification, nontoxicity, surfaces functionalities for colloidal stabilities, targets distribution, GNPs had received most attention as an X-ray's contrasting agent. Low-molecular-weight vascular contrasting age agents, like iodinates compounds, are common. These iodinated aromatics have a high-water solubility, indicating minimal toxicity. However, the period of blood circulation is brief, and waste is quickly removed by the kidneys. As a result, a limited imaging windows might necessitate numerous injections, increasing risks of thyroid-gland dysfunctions.

#### 5.1.3. Antibacterial Activity

Gold nanoparticles are able to inhibit bacterial growth by conferring themselves onto the bacterial cell surface due to their surface changes. Alteration of surface releases reactive oxygen species which causes protein denaturation, DNA destruction, and mitochondrial disfunction and finally leads to cell death [139]. A study reported synthesis of gold nanoparticles using *Mentha piperita* and evaluated its antibacterial effect against *E. coli* and *S. aureus* and found that gold nanoparticles showed antibacterial activity against *E. coli* only [140]. Another study reported synthesis of gold nanoparticles using *Commelina nudiflora* and found that it was effective against *Salmonella typhi* and *Enterococcus faecalis* [141]. Abdel-Raouf et al. [110] reported synthesis of gold nanoparticles using Galaxaura elongate and evaluated its antibacterial activity against *Escherichia coli*, *Klebsiella pneumoniae*, *Staphylococcus aureus*, and *Pseudomonas aeruginosa* and MRSA.

### 5.2. Environmental Application

#### 5.2.1. Removal of Pollutants

GNP-based technologies are being developed now for pollution control and water purification in the environment. Bimetallic gold-palladium nanoparticles have been found to be a potent catalyst for degrading trichloroethene (TCE), which is one of the primary contaminants in groundwater, into a nontoxic form [142]. GNPs in water purifications system have been shown to effectively gather and eliminate halocarbon-based pollutants from drinking water [143] and improve mercury oxidation from coal-fired power plants [144].

#### 5.2.2. Ornamental Applications

GNPs were developed to selectively oxidize biomass-derived chemicals such as furfurals or hydroxymethyl furfurals to produce methyl-esters, carbon monoxide (CO), or trimethylamine. These chemicals are used in polymers and industrial solvents, as well as in flavour and fragrance applications [145]. A range of gases, including carbon monoxide (CO) and nitrogen oxides, have been detected using Au nanoparticle-based gas sensors (NOx) [146].

#### 5.2.3. Removal of Inorganic Compounds

Green GNPs are widely recognised for their catalytic activity, particularly their catalytic reduction abilities. Although gold is not commonly used as a catalyst, gold nanoparticles have been reported to decrease ferrocyanide (III), nitroarenes, cyanosilylation of aldehydes, and deoxygenation of epoxides into alkenes. For example, p-nitrophenols, which are common by-products of the production of herbicides, pesticides, and synthetic dyes and are known to be environmentally poisonous and inhibitory in nature, have been successfully reduced to p-amino phenols by green synthesized GNPs, which would otherwise be incapable of being converted to its neutral and nontoxic form even by the strongest reducing agent [147–149].

## 6. Future Perspective

Nanotechnology is a rapidly expanding area with several applications in various fields. Gold nanoparticles are synthesized using a variety of processes because of their vast range of uses. Traditional chemical procedures have limitations, either in the form of chemical contamination during the synthesis process or in future applications. Chemical reduction of gold uses a variety of chemicals (reducing agents) that are usually hazardous and difficult to dispose of owing to environmental concerns. Synthesis is also carried out at higher temperatures in a variety of different situations, which generate a lot of heat and are highly expensive. Biological synthesis of gold nanoparticles has sparked considerable attention because it is a quick, ecofriendly, nonpathogenic, and cost-effective method that can be completed in a single step at room temperature and pressure. Compared to standard physical and chemical techniques, biological synthesis is an environmentally friendly approach that uses a diverse variety of resources such as plants, bacteria, actinomycetes, yeast, and fungi. The biosynthesis of gold nanoparticles is still in its early stages of investigation. There are a few issues that must be addressed. Several studies are still required to better understand the impacts of time, temperature, light, and other elements on the formation of gold nanoparticles, as well as the control of the nanoparticle size and shape. Furthermore, researchers face challenges due to a lack of knowledge of the chemical components and mechanisms involved in the reduction and stability of biosynthesized gold nanoparticles. As a consequence, more studies are recommended on the mechanism of gold nanoparticle synthesis and its influence on the shape and size of gold nanoparticles for various applications.

## 7. Conclusion

Biological approach for nanoparticle synthesis is an important alternative in the development of clean, nontoxic, cost-effective, and environmentally friendly technologies for the synthesis of GNPs, with substantial advantages over previous approaches. Many biological agents have the capacity to synthesise GNPs both inside and outside the cell. Research into the production of GNPs is still in its early stages. For widespread usage of GNPs in commercial applications, more research is required on biosynthesis processes and with well-defined size and shape. The capacity to vary the features of GNPs simply by changing their size or shape is intriguing, and it will be employed in unique applications in the future. GNPs are employed in a wide range of applications, including electronics and catalysis, as well as biology, medicine, and medical diagnostics and therapy. However, further research into the mechanics and kinetics of GNP production is required, since this might lead to process optimization, eventually leading to GNP synthesis with strict control over size, shape, and large-scale manufacturing.

## Figures and Tables

**Figure 1:** Synthetic methods for the synthesis of gold nanoparticles.

**Figure 2:** Mechanism of GNPs biosynthesis [22].

**Figure 3:** Green synthesis of GNPs from a plant [68].

**Table 1:** Bacteria synthesize gold nanoparticles.

Bacteria	Size (nm)	Shape	Reference
*Lyngbya majuscula*	20	Spherical	[35]
*Rhodopseudomonas capsulata*	10–20	Spherical	[31]
*Pseudomonas aeruginosa*	10–20	Spherical	[36]
*Pseudomonas denitrificans*	30–35	Face-centred cubic	[37]
*Marinobacter pelagius*	15	Triangular, spherical, polygonal	[38]
*Stenotrophomonas* sp.	20–60	Multishaped	[39]
*Bacillus megaterium* DO1	1.8 ± 0.9	Spherical	[40]
*Lactobacillus* sp.	30–60	Hexagonal	[41]
*Geobacillus stearothermophilus*	13	Polydisperse, circular	[42]
*Thermomonospora* sp.	8–13	Spherical	[43]
*Arthrobacter* sp. 61B	8–40	Spherical	[44]
*Bacillus subtilis*	7.3–7.6	—	[45]
*Stenotrophomonas maltophilia*	40	Oval	[46]
*Paracoccus haeundaensis* BC74171 T	20.93 ± 3.46	Spherical	[47]

**Table 2:** Fungi synthesize gold nanoparticles.

Fungus	Size (nm)	Shape	Reference
*Colletotrichum* sp.	30–50	Decahedral or icosahedral	[54]
*Fusarium oxysporum*	128 ± 70	Aggregates	[55]
*Helminthosporium solani*	3–80	Polydispersed extracellularly	[56]
*Neurospora crassa*	34	Spherical	[57]
*Penicillium brevicompactum*	20∼60	Spherical	[58]
*Trichoderma koningii*	40–50	Smaller spheres to polygonal spheres	[59]
	10–14		
*Verticillium* sp.	30 ± 9	Spherical	[60]
*Verticillium luteoalbum*	<20	Spherical	[61]
*Cylindrocladium floridanum*	19.05	Spherical	[62]
*Phanerochaete chrysosporium*	20–110	Spherical	[63]
*Volvariella volvacea*	30–150	Spherical	[64]
*Pichia jadinii*	<110	Spherical	[65]
*Yarrowia lipolytica*	9–27	Spherical	[66]
*Candida albicans*	20–40	Spherical	[67]

**Table 3:** Plants synthesize gold nanoparticles.

Plant	Size (nm)	Part of plant used	Reference
*Sapindus mukorossi*	9–19	Fruit pericarp	[74]
*Prunus domestica*	13–27	Fruit	[75]
*Magnolia kobus*	5–300	Leaf	[71]
*Diospyros kaki*	15–400	Leaf	[71]
*Coleus amboinicus lour*	8.0–31.8	Leaf	[76]
*Cassia auriculata*	25–35	Leaf	[77]
*Abelmoschus esculentus*	55–85	Seed	[78]
*Zingiber officinale*	15–25	Root	[78]
*Rosa hybrid*	10	Petals	[79]
*Nyctanthes arbortristis*	19.8	Flower extract	[80]
*Gnidia glauca*	50–150	Flower extract	[81]
*Salicornia brachiata*	22–35	Plant	[82]
*Soursop*	16	Fruit	[83]
*Sphaeranthus indicus*	25	Leaf	[84]
*Stachys lavandulifolia*	56.3	Plant	[85]
*Sterculia acuminata*	6.9–26.6	Fruit	[86]
*Stevia rebaudiana*	5–20	Leaf	[87]
*Syzygium cumini*	13–30	Seed	[88]
*Terminalia chebula*	6–60	Plant	[89]
*Thymus vulgaris*	35	Plant	[90]
*Trigonella foenum-graecum*	15–25	Seeds	[91]
*Zingiber officinale*	5–15	Plant	[92]
*Zostera noltii*	26 ± 6	Plant	[93]
*Mariposa christia vespertilionis*	50–70	Leaf	[94]
*Nepenthes khasiana*	50–80	Leaves	[95]
*Nerium oleander*	2–10	Leaf	[96]
*Nyctanthes arbor-tristis*	19.8 ± 5.0	Flower	[80]
*Nymphaea nouchali*	54.7	Leaf	[97]
*Opuntia ficus-indica*	5	Plant	[98]
*Garcinia indica*	20 and 30	Fruit	[99]
*Ginkgo biloba*	10–40	Leaf	[100]
*Hibiscus sabdariffa*	7 ± 2	Leaf	[101]

**Table 4:** List of biomolecules involved in the production of GNPs.

Biomolecules	Types	Sizes (nm)	Reference
Linoleic acids	Fatty acids	20	[112]
Tannic acids	Fatty acids	9–12	[113]
NADPH-dependent enzymes	Enzymes	26	[114]
Amino-dextran	Polysaccharides	19–40	[115]
Chitosan	Polysaccharide	—	[116]
Glucose	Carbohydrate	22–38	[117]
Sucrose	Carbohydrate	4–16	[117]
Raffinose	Carbohydrate	30–48	[117]
Dextrose	Carbohydrate	25, 60, 120	[118]
Starch	Polysaccharide	11–15	[119]
Bovine serum-albumin	Proteins	—	[120]
Serrapeptase	Proteins	20–200	[121]
Trypsins	Enzymes	—	[122]
Glycosaminoglycans	Mucopolysaccharides	—	[123]
Serratiopeptidase	Enzymes	—	[124]
DNA's	Nucleotides	45–80	[125]
Aspartates	Amino acids	30	[126]
Phospholipids	Lipid	5	[127]

## Data Availability

All data used to support the findings of this study are included within the article.
